The article "Dimethyl Fumarate Ameliorates Nucleus Pulposus Cell Dysfunction through Activating the Nrf2/HO-1 Pathway in Intervertebral Disc Degeneration" was published in 2021. Journal: Comput Math Methods Med.

# Dimethyl Fumarate Ameliorates Nucleus Pulposus Cell Dysfunction through Activating the Nrf2/HO-1 Pathway in Intervertebral Disc Degeneration

**DOI:** 10.1155/2021/6021763

**Published:** 2021-10-31

**Authors:** Ruihong Wang, Dawei Luo, Zhiwei Li, Huimin Han

**Affiliations:** ^1^Department of Spine Surgery, Weifang People's Hospital, Weifang 261041, China; ^2^Department of Spine Surgery, Liaocheng People's Hospital, Liaocheng 252002, China

## Abstract

**Background:**

Oxidative stress, inflammation, and nucleus pulposus cells (NPCs) apoptosis are involved in pathogenesis of intervertebral disc (IVD) degeneration (IVDD). Dimethyl fumarate (DMF) has been found to effectively depress oxidative stress and inflammation via the Nrf2 pathway. Hence, this project was designed to explore the underlying mechanisms of how DMF protects NPCs from damage by LPS challenge.

**Methods and Results:**

CCK8 assay and flow cytometry of apoptosis indicated that DMF treatment attenuated LPS-induced NPC damage. Western blot analysis demonstrated that DMF enhanced the expressions of nuclear factor-erythroid 2-related factor 2 (Nrf2) and heme oxygenase-1 (HO-1) in LPS-challenged NPCs. DMF treatment significantly decreased the accumulation of ROS, downregulated inflammatory cytokines (p-NF-*κ*B, IL-1*β*, and TNF-*α*), and ER stress-associated apoptosis proteins (Bip, calpain-1, caspase-12, caspase-3, and Bax) in LPS-challenged NPCs. The level of antiapoptotic protein Bcl-2 was promoted by DMF treatment in LPS-challenged NPCs. Glutathione (GSH) assay showed that DMF treatment improved reduced to oxidized glutathione ratio in LPS-challenged NPCs. Furthermore, the results of western blot analysis indicated that in LPS-challenged NPCs, DMF treatment ameliorated the elevated levels of matrix degradation enzymes (MMP-13, aggrecanase 1) and type I collagen and the reduced levels of matrix composition (type II collagen and ACAN). However, Nrf2 knockdown abolished these protective effects of DMF.

**Conclusion:**

Our data suggested that treatment with DMF mitigated LPS-induced oxidative stress, inflammation, and ER stress-associated apoptosis in NPCs via the Nrf2/HO-1 signaling pathway, thus reliving LPS-induced dysfunction of NPCs, which offered a novel potential pharmacological treatment strategy for IVDD.

## 1. Introduction

Intervertebral disc (IVD) degeneration (IVDD) is considered the primary causative factor of low back pain, which bothers approximately 10% of people worldwide [1, 2]. IVD is constituted by a central nucleus pulposus (NP) and an outer annulus fibrosus (AF). The NP is a hydrophilic gelatinous structure and contains large quantities of proteoglycans, mainly composed of type II collagen (Col-II) and aggrecan (ACAN). The AF is a collagenous concentric lamellae made up of type I collagen (Col-I) [3]. It has been reported that, in IVDD, the matrix composition of ACAN and col-II is degraded by matrix metalloproteinases (MMPs) and aggrecanases then replaced by Col-I, which leads to functionally disability of IVD [4].

Although the pathogenesis of IVDD is unclear yet, oxidative stress, inflammation, and nucleus pulposus cell (NPC) apoptosis play vital roles in disc degeneration [5]. The bulk of reactive oxygen species (ROS) generated during oxidative stress could directly impair NPCs and increase the expression of MMPs to degrade the IVD matrix [6, 7]. Wang et al. have shown that the increased expression of inflammatory cytokines, such as tumor necrosis factor-*α* (TNF-*α*) and interleukin-1*β* (IL-1*β*), accelerated the process of IVDD by inducing ACAN degradation [8]. And the excessive apoptosis of NPCs causes a reduced synthesis of the matrix, which further leads to the degeneration of intervertebral disc [9]. Therefore, the best way for IVDD therapy is to inhibit the oxidative stress, inflammation, and excessive apoptosis of NPCs.

The endoplasmic reticulum (ER), as an organelle for protein synthesis, signal transduction, and dynamic Ca^2+^ storage, plays an important role in determining cell fates [10]. Various conditions, such as hypoxia, starvation, inflammation, Ca^2+^, and redox imbalance, can affect the functions of the ER, leading to the so-called ER stress [11]. Generally, prolonged ER stress causes the activation of the proapoptotic pathway, which leads to the pathogenesis of many diseases [12]. Studies have demonstrated that the excessive and persistent ER stress involves inflammation and cell apoptosis pathways, thus leading to the matrix degradation and NPCs apoptosis in intervertebral disc [13, 14]. But the detailed mechanism was not clear yet. Caspase-12 is a proapoptotic protease located on the outer surface of the ER membrane, which is activated by calpain, an intracellular Ca^2+^-dependent cysteine protease [15–17]. Increased ROS concentration in the ER promotes the opening of Ca^2+^ channel, and Ca^2+^ enters cytoplasm, subsequently stimulates calpain protease, cleaves caspase-12, and activates the apoptosis pathway [17]. Hence, we speculated that LPS induced ER stress-apoptosis in NPCs through calpain-caspase-12 dependent pathway.

Dimethyl fumarate (DMF), as a well-known agonist of nuclear factor-erythroid 2-related factor 2 (Nrf2) responsive genes [18], has always been used as drugs in various degenerative diseases. For instance, DMF contributes to diabetic wound healing through activating Nrf2 and suppressing downstream inflammation [19]. Nrf2 plays an important role in antioxidative stress via promoting the expressions of several antioxidative genes, such as heme oxygenase-1 (HO-1) and NADPH quinone oxidoreductase-1 (NQO-1) [20–22]. Furthermore, Nrf2 can confer adaptive protection against inflammation to maintain cellular homeostasis, thus easing the subsequent downstream proapoptotic pathways [23, 24]. It was shown that activation of Nrf2 repressed oxidative stress-mediated ER stress, mitochondrial dysfunction, and apoptosis in septic liver injury [25]. However, the relationship between Nrf2, ER stress, and apoptosis in IVDD has not been elucidated until now.

In this research, we assessed the capability of DMF to improve IVDD by inducing oxidative stress, inflammation, and ER stress-associated apoptosis in NPCs using lipopolysaccharides (LPS) and explored the involvement of possible related signaling pathways. Our results presented that DMF could significantly relieve oxidative stress and inflammation in LPS-induced NPCs via the Nrf2/HO-1 pathway. Importantly, we found that DMF could also inhibit ER stress-mediated apoptosis through the Nrf2/HO-1 signaling pathway. These findings improve our understanding of the underlying mechanisms by which DMF attenuates IVDD and provides new ideas for IVDD therapeutic strategy.

## 2. Material and Methods

### 2.1. Cell Culture and Treatment

Human NPCs were purchased from ScienCell Research Laboratories (4800, ScienCell, Texas, USA) and cultured in Nucleus Pulposus Cell Medium (NPCM, ScienCell, Texas, USA) in an incubator with 5% CO_2_ at 37°C. The medium was changed every two days, and the cells were subcultured when the confluence reached 90%~95%. The cells were subcultured for 2~3 passages before the subsequent experiments. LPS and DMF were purchased from Sigma-Aldrich (Darmstadt, Germany) and stocked in PBS solution at -20°C. Cells were cultured in fresh medium for 6 hours, then stimulated with varying concentrations of LPS (0, 0.4, 0.8, 1.2, and 2.0 *μ*g/ml) to establish the NP cell injury model. Similarly, NPCs were treated with DMF at gradient concentrations of 0, 10, 20, 50, 100, and 200 *μ*M. After treatment with LPS or DMF for 24 h, 48 h, and 72 h, the CCK8 assay was executed to evaluate the cell viability.

### 2.2. Cell Viability (CCK-8) Assay

Approximately 2 × 10^5^/well of NPCs were seeded into 96-well plates. Following different treatment for 24 h, 48 h, and 72 h, the viability was tested by the CCK-8 kit (MedChemExpress, New Jersey, USA). In details, the cells were cultured in NPCM containing 10% CCK-8 solution for 2 hours and then tested optical density (OD) value at 450 nm using a Gen5 microplate reader (BioTek, Vermont, USA). The NP cells without treatment served as control.

### 2.3. Measurement of ROS Production

The intracellular ROS was evaluated by the DCFDA cellular ROS detection assay kit (Abcam, Cambridge, UK). The treated NP cells (2 × 10^5^/well) were seeded at cell slides and incubated for 48 h. Then, these cell slides were incubated with 10 *μ*M ROS working solution at 37°C for 45 min. Next, cell slides were washed with PBS. The intracellular ROS was measured under a fluorescence microscope (Leica DMI 3000B, Germany). The fluorescence intensity was analyzed by the ImageJ software version 8.0 (Bio-Rad, Hercules, USA).

### 2.4. Glutathione Assay

Relative changes in intracellular reduced glutathione (GSH) and oxidized glutathione (GSSG) levels were determined with the GSH/GSSG-Glo Assay kit (Promega, WI, USA). Briefly, the cells were collected and resuspended in HBSS buffer, then plated in a 96-well luminometer-compatible plate at 10,000 cells/well. 25 *μ*l of either total GSH lysis reagent or GSSG reagent was added to the wells and incubated at room temperature on a shaker for 5 min. Then 50 *μ*l of freshly prepared luciferin generation reagent was added to each well followed by 30 min incubation at room temperature. 100 *μ*l of luciferin detection reagent was then added to each well. After 15 min of incubation, luminescence was measured using a LUMIstar Omega Microplate Luminometer (BMG Labtech). Wells without cell and only HBSS buffer were used for background luminescence detection. Relative luminescence unit (RLU) for GSH levels was determined by subtracting RLU of GSSG from RLU of total glutathione. The ratio GSH/GSSG was calculated using the formula as follows.

(1) $$\begin{array}{c} \text{Ratio GSH}/\text{GSSG}=\frac{\mu \text{M total}-\left(\mu \text{M GSSG}\times 2\right)}{\mu \text{M GSSG}}. \end{array}$$

### 2.5. Western Blot

Total proteins were extracted by RIPA buffer (Beyotime, Shanghai, China) supplemented with PMSF (Beyotime, Shanghai, China). The protein concentration was measured by the BCA Protein Assay Kit (Thermo Fisher, Waltham, USA). Then, equal amounts of protein were loaded on 8–12% SDS-PAGE gels and transferred onto a PVDF transfer membrane (Millipore, Massachusetts, USA). After blocking with 5% skimmed milk solution, the membranes were incubated with specific primary antibodies overnight at 4°C followed by further incubation with the secondary antibody at room temperature for 2 h. Both primary and secondary antibodies were purchased from Thermo Fisher (Waltham, USA), including anti-*β*-actin, anti-Nrf2, anti-HO-1, anti-p-NF-*κ*B, anti-IL-1*β*, anti-TNF-*α*, anti-Bip, anti-calpain-2, anti-active caspase-12, anti-active caspase-3, anti-Bax, anti-Bcl-2, anti-ACAN, anti-Col-II, anti-Col-I, anti-MMP-13, anti-aggrecanase 1, and secondary antibody IgG. Finally, the protein bands were detected using the ECL Plus Reagent (Thermo Fisher, Waltham, USA), and their densitometry was analyzed with the ImageJ software version 8.0(Bio-Rad, Hercules, USA). With *β*-actin as control, the expression of total protein was normalized.

### 2.6. Flow Cytometry Analysis of Apoptosis

The cell apoptosis rate was evaluated using the Annexin V-FITC/PI Apoptosis Detection kit (Vazyme Biotech, Nanjing, China). Briefly, the cells were seeded into 6-well cell culture plates (4 × 10^5^ cells/well). After various treatments, the cells were collected, washed with PBS, and resuspended in 500 *μ*l binding buffer. Then, 5 *μ*l Annexin V-FITC and 5 *μ*l PI staining solution were added to the buffer, gently shaken, and incubated at room temperature for 10 min in the dark. Cells were analyzed by flow cytometry (Beckman Coulter, California, USA) within 1 h.

### 2.7. Transfection of shRNA

The shRNA lentivirus plasmids for human Nrf2 (sh-Nrf2, Santa Cruz Biotechnology, USA) and control shRNA Plasmid-A (sh-NC, Santa Cruz Biotechnology, Delaware, USA) were transfected into NPCs using Lipofectamine LTX Reagent with Plus Reagent (Thermo Fisher, Waltham, USA). The knockdown efficiency of sh-Nrf2 was confirmed by western blot and RT-qPCR.

### 2.8. RT-qPCR

Total RNA was collected using TRIzol Reagent (Takara, Japan). 1 *μ*g of RNA was collected as a template and reversely transcribed using PrimeScript™ RT Master Mix (TaKaRa, Japan). The reversed cDNAs were used for the following RT-qPCR experiments using the SYBR®Green kit (TaKaRa, Tokyo, Japan), and the reactions were performed using an ABI 7500 Sequencing Detection System. The primers used in RT-qPCR were synthesized by GENEWIZ (Suzhou, China). The primer sequences are displayed in Table 1. With GAPDH as a reference gene, Ct and 2^−*ΔΔ*Ct^ values were employed to calculate the mRNA levels.

### 2.9. Statistical Analysis

All data were collected from three independent experiments and presented as mean ± SD. Statistical analyses were carried out using GraphPad Prism8 (GraphPad Software, Inc.). Differences among groups were evaluated using one-way ANOVA. Differences in data between each group were further analyzed by Sidak's multiple comparisons test, and mean differences were expressed with 95% confidence intervals. *P* values < 0.05 were considered statistically significant differences and displayed in the figures as ^∗^. *P* values < 0.01 are shown as ^∗∗^, and <0.001 as ^∗∗∗^, respectively.

## 3. Results

### 3.1. DMF Increased Cell Viability in LPS-Induced NPCs

Here, we used LPS challenge with gradient concentrations (0, 0.4, 0.8, 1.2, and 2.0 *μ*g/ml) to establish an *in vitro* cell model of degenerative NPCs. The results demonstrated that the viability of NPCs was impeded in a dose-dependent manner, and a remarkable injury was displayed on LPS-challenged NPCs compared to control (0 *μ*g/ml) when the concentration was up to 1.2 *μ*g/ml (Figure 1(a)). Therefore, we chose the LPS concentration of 1.2 *μ*g/ml to stimulate NPCs for the following experiments, establishing a degenerative NPCs model.

Before comparing the cytoprotective effect on the degenerative NPCs, the dose-dependent cytotoxic effect of DMF was measured by the CCK-8 assay. The results demonstrated that 10-100 *μ* MDMF is not toxic to NPCs and the cell viability was markedly increased within the 10-50 *μ*M DMF treatment (Figure 1(b)). Later, the reversed effect of DMF on LPS-induced NPCs injury was measured.  Figure 1(c) indicates that DMF relieved the NPC viability reduction aroused by LPS in a dose-dependent manner. Notably, the NPC viability was almost consistent with the control group when DMF concentration was 50 *μ*M, suggesting that DMF treatment effectively reversed LPS-induced cell damage. Thus, we chose 50 *μ*M DMF as the rescued concentration for LPS-challenged NPCs.

### 3.2. Nrf2/HO-1 Pathway Was Involved in Improving Cell Viability of LPS-Challenged NPCs

To further explore how DMF protect LPS-challenged NPCs against cell damage, the western blot analysis was applied to detect the level of Nrf2 and its downstream effector HO-1.  Figure 2(a) indicated that LPS administration inhibited Nrf2 and HO-1 expression, while its level recovered to a large extent upon DMF treatment. Subsequently, the specific shRNA of Nrf2 was used to further confirm the role of Nrf2/HO-1 in degenerative NPCs. First of all, the knockdown efficiency of Nrf2 shRNA was detected by RT-qPCR and western blot, and the mRNA level of Nrf2 was decreased 80% and the expression level of Nrf2 was decreased 85% (Figure 2(b)), which meant it was an available specific shRNA for Nrf2 knockdown. As shown in Figure 2(c), Nrf2 knockdown abolished the upregulated expression of HO-1 by DMF treatment in LPS-challenged NPCs. This suggested that HO-1 did work downstream of Nrf2. Moreover, the NPCs viability was determined using the CCK-8 assay under Nrf2 knockdown.  Figure 2(d) displayed the viability of LPS-challenged NPCs was increased with DMF treatment, while Nrf2 knockdown significantly attenuated the protective effect of DMF to LPS-challenged NPCs. These results suggested that DMF exerted a protective role on degenerative NPCs via triggering the Nrf2/HO-1 pathway.

### 3.3. DMF Ameliorated LPS-Induced Oxidative Stress and Expression of Inflammatory Cytokines in NPCs

Under oxidative stress, excessive amounts of ROS generation promote the process of disc degeneration [26]. As illustrated in Figure 3(a), ROS accumulation in NPCs markedly increased following LPS induction compared with the control group, while DMF treatment decreased ROS production by LPS challenge. Nrf2 knockdown reversed the elevated production of ROS in LPS-challenged NPCs. Glutathione (GSH) is thought to be critically important in protecting the cells from ROS production. Hence, we determined the intracellular GSH formation by assessing the ration of reduced glutathione (GSH) to oxidized glutathione (GSSG) in NPCs with a luminescence-based assay (Figure 3(b)). The results displayed that DMF significantly improved while LPS challenge notably reduced the ratio of GSH/GSSG. And DMF markedly reversed the reduced ratio of GSH/GSSG caused by LPS challenge in NPCs. However, Nrf2 knockdown counteracted this reversed effect of DMF in LPS-challenged NPCs.

In response to oxidative stress, a series of inflammatory cytokines were secreted by NPCs. Therefore, western blot was executed to determine the expressions of p-NF-*κ*B, IL-1*β*, and TNF-*α*. As indicated in Figure 3(c), the expressions of p-NF-*κ*B, IL-1*β*, and TNF-*α* were decreased by DMF compared with the LPS group. Similarly, the levels of these inflammatory cytokines were recovered under Nrf2 knockdown (Figure 3(c)). These results suggested that DMF attenuated LPS-induced oxidative stress and inflammation in NPCs via the activation of the Nrf2/HO-1 pathway.

### 3.4. DMF Ameliorated ER Stress-Mediated Apoptosis in LPS-Challenged NPCs

ER stress is one of the main causes of NPC apoptosis. Here, we demonstrated that DMF treatment reduced the increased level of ER stress marker Bip in LPS-challenged NPCs (Figure 4(a)). However, Nrf2 knockdown reversed the enhanced expression of Bip by LPS challenge in NPCs. This suggested that DMF treatment suppressed ER stress induced by LPS through the Nrf2/HO-1 pathway.

Generally, excessive or prolonged ER stress will trigger cell apoptosis. The outcomes of western blot illustrated that the expressions of active caspase-3 and Bax were promoted, while the level of Bcl-2 was diminished in LPS-challenged NPCs compared with the control group (Figure 4(b)). Calpain-2 is implicated in caspase-12 activation dependent on Ca^2+^ flux under ER stress [27]. Our results indicated that the expressions of calpain-2 and active caspase-12 were increased in LPS-challenged NPCs compared with the control group (Figures 4(a) and 4(b)). This illustrated that LPS induced ER stress-mediated apoptosis through the calpain-2/caspase-12-dependent pathway in NPCs, thus leading to NPC apoptosis and subsequently disc degeneration. Nevertheless, treatment with DMF decreased the levels of calpain-2, active caspase-12, active caspase-3, and Bax and increased the level of Bcl-2 in LPS-challenged NPCs. These effects of DMF were reversed by Nrf2 knockdown (Figures 4(a) and 4(b)), which suggested DMF attenuated ER stress-mediated apoptosis in LPS-challenged NPCs via activating the Nrf2/HO-1 pathway. The flow cytometry of cell apoptosis was executed to further confirm the effect of DMF on ER stress-mediated apoptosis (Figure 4(c)), and the data were consistent with western blot.

### 3.5. DMF Alleviated LPS-Challenged NPCs Dysfunction

Oxidative stress, inflammation, and ER stress-mediated apoptosis are cooperative in IVDD progression. In degenerative disc, the syntheses of proteoglycans (ACAN, Col-II) were decreased, and the expressions of matrix metalloproteinases (MMPs) and aggrecanases were increased to promote the matrix degradation; then proteoglycans were replaced by Col-I. In our study, the levels of MMP-13, aggrecanase 1, and Col-I were enhanced, while the levels of ACAN and Col-II were decreased in LPS-challenged NPCs compared with the control group. DMF treatment decreased the levels of MMP-13, aggrecanase 1, and Col-I but increased the levels of ACAN and Col-II. However, these effects were also reversed by Nrf2 knockdown (Figure 5).

## 4. Discussion

The current management of IVDD is only able to relieve the symptoms but do not solve the underlying pathology of degeneration. In the clinical treatment, growth factors or proteinase inhibitor injected into IVDD tissues are applied to the early IVDD but with a limited therapeutic effect [28], while the operation is used to relieve nerve compression in late IVDD but helpless for the recovery of IVDD [29]. Hence, a better strategy is needed.

In the current study, we investigated whether DMF could attenuate the degeneration of NPCs. The results showed that the protective mechanism of DMF was related to the activation of the Nrf2/HO-1 signaling pathway which mitigates LPS-induced oxidative stress, inflammation, and ER stress-mediated apoptosis in NPCs. It might be a novel therapeutic option that could be used to mitigate disc degeneration.

The Nrf2/HO-1 pathway, the principal cellular defense system of antioxidative stress and anti-inflammatory response, plays an indispensable role in protecting intervertebral disc from degeneration [24, 30, 31]. DMF, the Nrf2 activator, is applied to the treatment of multiple sclerosis and psoriasis [32, 33]. Oxidative stress not only enhances matrix degradation and inflammation but also promotes apoptosis of viable and functional cells in the microenvironment of IVDs [34]. Many antioxidative drugs, such as aspirin, fullerol, and berberine, are used to ameliorate ROS in IVDD [26, 35, 36]. It is demonstrated that DMF activated Nrf2 to stimulate the production of glutathione (GSH), which is the most important scavenger of ROS [33], hence, to protect the cells against ROS-induced cytotoxicity. Here, we indicated that DMF decreased the production of ROS by activating the Nrf2/HO-1 signaling pathway. We also observed the increased GSH production in DMF-treated NPCs, thereby eliminating excessive ROS production in LPS-challenged NPCs by activating the Nrf2/HO-1 signaling pathway. Nicolay et al. demonstrated that DMF downregulated NF-*κ*B in cutaneous T-cell lymphoma cells, restored the apoptosis sensitivity, and inhibited tumor growth [37]. Our study suggested that DMF also downregulated the expression of p-NF-*κ*B in LPS-challenged NPCs. Nuclear translocation of NF-*κ*B initiates the transcription of inflammatory cytokines. Importantly, both TNF-*α* and IL-1*β* upregulate the expressions of matrix degrading MMPs and two major aggrecanases (ADAMTS-4 and ADAMTS-5) in NPCs [38, 39]. In our study, the expression of proinflammatory cytokines (IL-1*β*, TNF-*α*), MMP-13, and aggrecanase 1 were increased in LPS-challenged NPCs. DMF downregulated the expression of proinflammatory cytokines, both IL-1*β* and TNF-*α*, in LPS-challenged NPCs via activating the Nrf2/HO-1 signaling pathway, thereby downregulating the expressions of MMP-13 and aggrecanase 1, reducing the matrix compositions of Col-II and ACAN degradation and ameliorating the process of IVD deterioration.

It does rely on ER function by which the NPCs produce extracellular matrix to ensure that the tissue can better withstand enhanced hydrostatic pressure and maintain the normal function of NP [40]. As the IVDD processes, the ER-related chaperon protein Bip was upregulated in the disc [13, 41]. Here, we also indicated that the expression of Bip increased in LPS-challenged NPCs. Persistent ER stress has been demonstrated to be associated with NPC apoptosis in IVDD, leading to decreased NPC number and subsequently decreased synthesis of the disc matrix, but the underlying mechanism remained elusive. The report demonstrates that impaired Ca^2+^ homeostasis plays an essential role in glycation end product- (AGE-) mediated ER stress and subsequent apoptosis in NPCs [42]. In this study, we revealed that Ca^2+^-dependent protease calpain-1 was increased in LPS-challenged NPCs. Furthermore, the activity of its downstream effector caspase-12 and proteins related to apoptosis (caspase-3, Bax) was also increased by LPS induction. DMF treatment reduced these elevated levels in LPS-challenged NPCs due to the activation of the Nrf2/HO-1 pathway. This suggested that DMF treatment ameliorated LPS-induced ER stress-mediated apoptosis dependent on the calpain-1/caspase-12 pathway, thus reversing its impairment on NPCs in the intervertebral disc. Consequently, the NPC apoptosis rate and the degradation of the disc matrix (Col-II, ACAN) were also reduced by DMF treatment. Our study provides a new thought for the mechanisms of ER stress-mediated apoptosis in IVDD.

The conclusion in the current study is drawn based on the *in vitro* results. Although the human NPCs derived from the intervertebral disc were used to mimic the *in vivo* conditions to some extent, LPS treatment differed from the actual physiological or pathological conditions. Besides, the impairment of IVD of oxidative stress and inflammation-mediated apoptosis was studied extensively, but the detailed mechanisms of ER stress-mediated apoptosis were not clear yet. Here, we demonstrated LPS induced ER stress-mediated apoptosis dependent on the calpain-1/caspase-12 pathway in degenerative NPCs. The roles of other branches of ER stress in mediating apoptosis still need to be further explored in the IVDD process.

## 5. Conclusion

In conclusion, we demonstrated that DMF effectively relieved oxidative stress, inflammation, and ER stress-associated apoptosis via activating the Nrf2/HO-1 signaling pathway, ameliorating the process of IVDD *in vitro*, which might be a potential novel target for the IVDD therapy.

## Figures and Tables

**Figure 1:** Determination of DMF function on LPS-stimulated NPCs. NPCs were treated with different concentrations (0, 0.4, 0.8, 1.2, and 2.0 *μ*g/ml) of LPS (a), gradient concentrations (0, 10, 20, 50, 100, and 200 *μ*M) of DMF (b), and NPCs were pretreated with DMF (0, 10, 20, and 50 *μ*M) for 3 h and then stimulated by 1.2 *μ*g/ml LPS for 0, 24, 48, and 72 h (c). The cell viability was detected by the CCK-8 assay. Data are presented as mean ± SD (*n* = 3 per group).

**Figure 2:** DMF inhibits LPS-induced NPCs damage via activating the Nrf2/HO-1 pathway. (a) The Nrf2 and HO-1 expression was detected by western blot. (b) The negative control shRNA (sh-NC) and specific shRNA of Nrf2 (sh-Nrf2) were transfected into NPCs, respectively. The Nrf2 and HO-1 expression was detected by western blot and RT-qPCR. (c, d) The sh-NC and sh-Nrf2 were transfected into NPCs, respectively. After incubation for 36 h, the cells were treated with 50 *μ*M DMF for 3 h and then stimulated by 1.2 *μ*g/ml LPS. The Nrf2 expression was detected by western blot. Cell viability was detected by CCK-8 assay. Data are presented as mean ± SD (*n* = 3 per group). Differences among groups were evaluated using one-way ANOVA and followed by Sidak's multiple comparisons test between each group. ^∗^ is for *p* < 0.05, ^∗∗^ for *p* < 0.01, and ^∗∗∗^ for *p* < 0.001.

**Figure 3:** DMF decreases the production of ROS and the levels of inflammatory cytokines via the Nrf2/HO-1 pathway. (a) Fluorescence images show ROS levels in different groups. Scale bar: 100 *μ*m. The relative fluorescence intensity of ROS as control was analyzed by the ImageJ software. (b) The intracellular redox state of cell samples as indicated treatment was determined by measuring intracellular glutathione concentration and showed as the ratio of GSH/GSSG. (c) The expressions of p-NF-*κ*B, IL-1*β*, and TNF-*α* were detected by western blot. The densitometry of protein bands relative to control was analyzed by the ImageJ software. Data are presented as mean ± SD (*n* = 3 per group). Differences among groups were evaluated using one-way ANOVA and followed by Sidak's multiple comparisons test between each group. ^∗^ is for *p* < 0.05, ^∗∗^ for *p* < 0.01, and ^∗∗∗^ for *p* < 0.001.

**Figure 4:** DMF suppresses ER stress-mediated apoptosis in NPCs via activating the Nrf2/HO-1 pathway. (a) The NPCs were treated as the indicated treatment, and the level of ER stress (Bip, calpain-2) was detected by western blot. (b) The expressions of apoptosis-related proteins (caspase-12, caspase-3, Bax, and Bcl-2) were detected by western blot. The densitometry of protein bands relative to control was analyzed by the ImageJ software. (c) The NPC apoptosis rate under different treatments was detected by flow cytometry. Data are presented as mean ± SD (*n* = 3 per group). Differences among groups were evaluated using one-way ANOVA and followed by Sidak's multiple comparisons test between each group. ^∗^ is for *p* < 0.05, ^∗∗^ for *p* < 0.01, and ^∗∗∗^ for *p* < 0.001.

**Figure 5:** DMF alleviates the NPC degradation via activating the Nrf2/HO-1 pathway. The expressions of CCL3, MMP-2, aggrecanase 1, Col-I, ACAN, and Col-II were detected western blot. The densitometry of protein bands relative to control was analyzed by the ImageJ software. Data are presented as mean ± SD (*n* = 3 per group). Differences among groups were evaluated using one-way ANOVA and followed by Sidak's multiple comparisons test between each group. ^∗^ is for *p* < 0.05, ^∗∗^ for *p* < 0.01, and ^∗∗∗^ for *p* < 0.001.

**Table 1:** RT-qPCR primer sequences.

Gene name	Description	Primer sequence (5′-3′)
GAPDH	Forward	TGACGTGCCGCCTGGAGAAAC
	Reverse	CCGGCATCGAAGGTGGAAGAG
Nrf2	Forward	TACTCTGCTCGTATTGGCTGC
	Reverse	GGAGGAACTTCGTGTTCGATG

## Data Availability

The datasets used and/or analyzed during the current study are available from the corresponding author on reasonable request.

## Abbreviations

ACAN: Aggrecan
AF: Annulus fibrosus
Col-I: Type I collagen
Col-II: Type II collagen
DMF: Dimethyl fumarate
ER: Endoplasmic reticulum
FBS: Fetal bovine serum
GSH: Glutathione
HO-1: Heme oxygenase-1
IL-1*β*: Interleukin-1*β*
IVD: Intervertebral disc
IVDD: Intervertebral disc degeneration
LBP: Low back pain
NP: Nucleus pulposus
NPCM: Nucleus pulposus cell medium
NPCs: Nucleus pulposus cells
NQO-1: NADPH quinone oxidoreductase-1
Nrf2: Nuclear factor, erythroid 2-like 2
OD: Optical density
ROS: Reactive oxygen species
TNF-*α*: Tumor necrosis factor-*α*.
